RETRACTED

# A Novel MG 2D Animation Design Method under the Perspective of Convergence Media Using Intelligent Design Technology

**DOI:** 10.1155/2022/2568690

**Published:** 2022-07-09

**Authors:** Juan Xu, Kai Liu, Yang Yuan

**Affiliations:** Institute of Art and Design, Nanjing Institute of Technology, Nanjing, Jiangsu 211167, China

## Abstract

The arrival of the 5G era, along with the gradual acceleration of information technology development, makes all kinds of new media gradually integrated into all corners of people's life, work, and study. Communication systems are breaking the original boundaries and moving toward communion. “Convergence Media” is a general term of new media which is built on modern network technology and integrates various media forms. In this context, animation design not only is limited to two-dimensional or three-dimensional creation, but also formed a new form of animation expression, namely, MG animation. For MG animation, with its simple artistic modeling elements and flexible rhythm, people have gained new cognition. When the Internet information is transmitted, MG animation can output a large number of dynamic images and text to people in a very short time, which is similar to the current mode of new media communication. It can make information more attractive and appealing with the visual performance of MG animation. In order to improve the quality and efficiency of animation, convergence media technology is applied to the drawing and production of animation. The emergence and continuous improvement of software such as AE, PR, and PS and other software have a strong compatibility and can fully meet our various requirements for MG animation production, thus bringing the audience a different kind of animation experience. AE, a common software for video production, can create a variety of striking visual effects with high efficiency and precision, with powerful effects control and millions of plug-ins to achieve a wide range of animation effects. High-quality video rendering supports resolutions from 4 × 4 to 30,000 × 30,000 pixels including high-definition television (HDTV). Therefore, in terms of animation production, we can choose to mainly use AE for production and rendering. In terms of drawing tools, PS is the software of choice, with no delay in drawing, dithering correction, selection, and other features which are quite outstanding, and has a great advantage in drawing lines and coloring. Based on this, this paper mainly explores the design and production cases of MG 2D animation from the new media perspective using the intelligent design technology. The animation designed by the method in this paper can also be used for medical treatment management or lesion display in the medical field.

RETRACTED

## 1. Introduction

Electronic press, Internet radio, mobile newspaper, mobile radio, Internet TV, mobile TV, and so on have become the way we access information nowadays. They have integrated various functions of different media, and this trend is gradually expanding. Undoubtedly, we are in the era of convergence media. In the era of trinetworks integration, the role played by MG animation is becoming more and more prominent, which has proposed higher requirements on its quality ability, innovation consciousness, and integration ability. We should stand in the overall situation, study the impact of media convergence on MG animation, and discuss how to transform, innovate, and develop traditional 2D animation in the context of media convergence with case design [1]. Based on the characteristics of new media and traditional media integration, the article points out the challenges faced by the current 2D animation, analyzes the ability quality of China's 2D animation creation, according to the changes in industry application standards, needs to improve for special speed requirements, user behavior preferences, and other directions, and gives the corresponding strengthening measures.

MG animation (the full English name: Motion Graphics) is directly translated as motion graphics or graphic animation. MG animation in this paper is mainly a kind of video art, which integrates graphic design, animation design, and film language, and its expression form is rich and diverse, with strong inclusiveness. Specifically, MG animation is between graphic design and animation design, and it uses the expression form of graphic design in visual performance while using the production means of animation in technology. Through the combination of the two designs, MG animation transforms static flat images and shapes into dynamic visual effects, attracting the public's attention with its unique expression form and becoming more and more popular in the market, injecting fresh blood into the animation industry [1]. In the market, MG animation is a kind of cultural communication media and art symbol, which takes on the function of cultural communication. Nowadays, with the rapid development of the cultural industry, the public has a more diversified understanding of the aesthetic taste of contemporary design, and the progress of technology has made many various design styles appear in front of the public one after another. The current MG animation industry is still in its infancy compared to other types of animation [2]. With the development of science and technology and the gradual strengthening of our country, there is a growing need for more excellent animated shorts, including MG animation, to convey the truth, goodness, and beauty in society and bring people spiritual education to promote the harmonious development of society.

RETRACTED

## 2. The Content of MG 2D Animation

This case design primarily focuses on describing the source of creativity, the completion of the script, the creation of the storyboard, the midterm animation production, and the postcomposition parts of the process of making this 2D animation short film. It also describes the content of the short film as well as the significance of the short film.

The emergence of MG animation has given people a new understanding of animation. In terms of production methods, MG animation is more concise and convenient, and has a high value to the market. While traditional graphic design is based on graphics, which is a static visual expression, MG animation is based on graphic design, supplemented by the basic production principles of animation to produce a section of graphic image deformation-based dynamic expression form. MG animation can be visually designed while allowing the animation to form more compelling graphic content through narrative choreography. This form of creation is far more attractive than ordinary static image expressions or textual narrative expressions. In Wikipedia, MG animation is explained as the use of video or animation technology to create motion or transformation of graphics, often combined with audio and used in multimedia design projects; through the electronic media technology equipment, it is very useful in distinguishing static graphics and graphics with motion characteristics. MG animation takes the movement of graphics and text as the main expression form. This new art form not only inherits and carries forward the advantages of traditional graphic design in terms of text, graphics, and color, but also combines the movement qualities of animation, which has unique artistic expression [3, 4].

The creation idea of MG 2D animation short film “Waiting” comes from the new crown epidemic that broke out in Wuhan, Hubei, at the end of 2019, and many touching stories happened in the fight against the epidemic. According to the background of this era and many real stories, by consulting a lot of information, the theme of this short film was determined as waiting, about the emotional problems of a long-distance couple before and after the epidemic. On the one hand, they want to be with each other; on the other hand, under the circumstances of the epidemic, they need to think about the country as people, facing the contradiction between devotion to the country and accompanying their loved ones. Faced with this issue of personal and national concern, both sides need to make a choice. At the end of the story, the two sides overcome the epidemic and the lovers are finally married.

RETRACTED

“Waiting” is a short animation film that runs between three and five minutes and is made in 2D. The animation production of the movie makes use of a wide array of animation approaches, most of which are accomplished through the use of the software programs PhotoShop, After Effects, and Premiere. For the purpose of production in the animation creating process, 2D animation software is utilized. A flat style animated short film on the topic of antiepidemic measures was created by our team with the assistance of a variety of 2D software and postsynthesis tools.

This case design combines plot setting and technical means to design a public welfare animation short film “Waiting” with the current background of the epidemic. In China, there are not many two-dimensional animated short films with the theme of fighting the epidemic, so the design of this animated short film is innovative in the current market. The technique used in the short film is to see the big picture from a small perspective and to represent the general public from the perspective of an ordinary person, which makes the animation more immersive and persuasive. The film also absorbed the advantages of other films, making the characters more vivid and easier to be accepted by the audience and bringing the audience closer to each other.

## 3. Intelligent Design of the Case

### 3.1. The Intelligent Design of Some Characters

This work is a 2D animated short film with the theme of public welfare. There are few 2D animated short films with the theme of fighting against epidemics in China, and the technique used is mainly to see the big picture in a small way, with the role of an ordinary person to represent the general public, which makes the animation more immersive and persuasive. This film also absorbs the advantages of other films to make the characters more vivid and easier to be accepted by the audience and to narrow the distance between the audience, as shown in Figures 1 and 2.

The creation of animated characters is a crucial but sometimes overlooked part of making an animated film. It is the foundation upon which the rest of the animation is built, and it also contributes significantly to the creation of the animation's aesthetic and the progression of the story's plot, which may convey the film's central theme. Additionally, the design and construction of the script, which combine the producer's inner thoughts and modern aesthetic notions, should be unified with the animation character modeling. This is because the script is the combination of the producer's inner thoughts and contemporary aesthetic concepts. As Li Guangsuo proposed in “Animation Character Design,” character design is a crucial part of the creation of the whole animation work, which carries the development of the storyline, the style of the work, and the development trend. Excellent character styling design is not limited to the animation performance itself, but becomes a typical cultural symbol with excellent styling design and unique performance in the animation film, which generates a wide audience influence and can make it produce cultural value and meaning independent of the animation work [5]. Therefore, in the character design of this animation short film, according to the technique of seeing the big in the small, taking the ordinary people around as the prototype, combining the basic principles of animation production, and considering the difficulty of production afterwards, the final decision was made on the styling settings of the male and female main characters.

RETRACTED

### 3.2. Intelligent Scene Design

The creation of animation scenes is an essential component of the animation production process. It serves as a necessary assurance for the style and character performance of the animation film, and it is also a condition for the achievement of success for the film. The many visual effects that are applied to animation sequences have a direct impact on the entire animation film. In addition, a well-designed scene may relate the feelings of the characters to the development of the story. It is of vital importance to both the emotional performance and the progression of the storyline over the whole piece [6].

MG animation has the characteristics of graphic design; that is, rich colors can make the picture more attractive; at the same time, MG animation has a distinctive style and advantages compared with traditional animation in terms of color matching. It does not have complex light and shadow relationship, more by simple color matching and full digital display, so that it shows a unique sense of modernity [7]. It should be noted that the color matching also determines to a certain extent the style of the whole animation short film and has a great influence on the expression of the theme intention. In the process of color design of this film, we need to focus on how to focus the audience's attention on the part we want to emphasize, and we should pay attention to the design of the background color to unify and not overwhelm the main. The bright-toned scenes give people a comfortable and relaxed feeling, which is suitable for the beginning and end of the play, as in Figure 3; the gray-toned scenes give people a depressed and tense feeling, which is more suitable for the middle part of the play when the epidemic breaks out, as in Figure 4. Color is a very important element of scene design, and when designing the scenes, while retaining the color of the objects themselves, it is also necessary to combine their own experience and in the scene design, while retaining the color of the object itself, we also need to combine our own experience and plot development to make some artistic processing to form a certain scene style, making the scene of the short film more vivid and rich in emotion.

RETRACTED

Unlike most hand-drawn 2D animations, the focus of the film is not on the characters, but on the scene construction and the rendering atmosphere. For this animation, I think the fluidity of the animation itself and the overall picture unity principle are more important, so I focused on the scene construction and animation for more in-depth thinking and set the main shape, picture tone, and style of the animation before drawing work. Generally speaking, we will first build the set scene according to the preliminary script and then draw several elements to determine the basic position to ensure the overall unity of the picture later. And after the overall style of the animation is established, the various detailed places in the whole picture can be perfected. After the art style and subcamera design are finished, we can enter the midterm creation process. MG animation mainly consists of simple geometric drawing, and good drawing skills and color matching skills can greatly enhance the overall visual experience [8, 9].

In terms of software use, we mainly use PS as the drawing tool and AE as the processing tool. As MG animation mostly uses graphic elements, in the production process, the graphics needed are usually drawn out in PS and then imported into the animation software for postprocessing and production. Scene drawing is mainly to realize the scenes drawn in the process of sub-scene script creation on the software, which also needs to be based on the text and the whole MG animation tone, drawing scene elements in PS and importing them into the animation software.

When designing the scenes, we need to consider many settings that match the overall style, so that there cannot be anything that does not match the overall atmosphere. To integrate all the scenes of the whole animation, the way we adopt in our short film is to integrate the small elements of each scene, such as flowers or backgrounds or falling leaves, and so on, and make these small elements unified in style and coordinated in color, so these small elements can be used throughout the whole animation that brings a harmonious aesthetic feeling, such as Figures 5–7, which can meet the aesthetic style of the picture and realize the overall feeling of the whole picture at the same time [10–12].

RETRACTED

### 3.3. The Process of Storyboard Drawing

To depict a paragraph of text using audiovisual language, we must consider camera movement, scene size, and scene transition at each level of the process, starting with the text script and going through the text storyboard and shot script design [13, 14]. Storyboard script design is the work scope of animation preproduction, which is the foundation of the entire animation production, and it is also the working blueprint of the finished animation; therefore it must be thoroughly thought out and planned during this phase. This is due to the fact that storyboard screenplay design is part of the work scope of animation preproduction. Because the animation used throughout the short film was developed based on the storyboard scenario, its value cannot be emphasized. It is linked to the general rhythm of animation, as well as camera movement, action design, scene sequences, and so on, and it is present throughout the animation production process. The storyboard is a visual representation of the word script, and its design has a direct impact on the overall effect of the animation short film. A successful animation short film cannot be isolated from the storyboard design since it will have a direct impact on the overall impression of the animation short film. During the process of making the storyboard draft for this animation short film, the main idea and setting of the short film as well as the limited level were taken into account, and after carefully watching a large number of outstanding works, the storyboard was changed over and over again in the parts of scenery use, camera movement, and camera switching. The goal was to show the charm of the story in the best way possible (see Figures 8 and 9).

### 3.4. Intelligent Animation Process

I need to utilize keyframes on the timeline to have an object fall from point A to position B and then bounce upwards [15]. As the animation process progresses, we must examine the application of motion laws. For instance, I would like an object to fall from point A to point B and then bounce back up. This landing place will be smoothed out by default, and as a result, the ball will travel at a steady speed even if the speed is not modified or adjusted. The landing point is defined as the place B where the ball lands. When combined with the law of animation, however, A to B is a process of falling while accelerating; when it reaches the point where it will land, the ball will reach its maximum speed; it will then suddenly bounce up; and when it approaches the position of A, its speed will drop to its lowest possible level. The distance between A and B and the amount of time the ball moves are the major elements that influence the quality of the animation, according to this guiding notion.

RETRACTED

Movement is at the heart of animation, which is fitting considering that animation is an art form that focuses on motion. It is vital to make the movement of the figure in an animation smooth and natural, according to particular standards, in order to make the animation vivid. Two fundamental components of animation are the use of points in time and spatial amplitude. Excellent animation shorts will go to the trouble of polishing the character's movement rule and dynamic space expression. This is done to ensure that the character's shape and character, as well as the story background, cooperate with each other. Furthermore, this is done to achieve a humorous effect through the use of language, soundtrack, songs, body movements, etc., so that the entire short film is harmonious and unified and has animation characteristics. In order to create characters that are more vibrant and vivid, it is important, while creating them, to properly exaggerate their features and boost their dynamic flexibility, as shown in Figure 10.

Due to the need of animation for character movement performance, whether it is three-dimensional animation modeling or two-dimensional animation modeling, we will generally use three-dimensional modeling. The character design of MG animation has unique visual characteristics compared with other animation character designs, unlike the all-around three-dimensional design; the design of MG animation is a flat design that integrates the graphic design. Therefore, MG animation has certain special characteristics, which can break the limits of the form when in motion, stretching, deformation, and redesign to enhance the expressive power of the work. Although MG animation is different from 3D animation and 2D frame-by-frame animation which have a rich history, the production still needs to be integrated into the character like traditional animation, fully understand the character, design the movement according to the character and psychological activity, as well as grasp and portray the dynamics, and exaggerate the degree and elastic change [14]; all these are the core work of animation production and need to be carefully considered, as in Figure 11.

The best way to accurately express the character's action language in MG animation is to film your own performance on a mobile phone video and use it as a reference. In addition, action performance footage from well-known movies and television series can be used. These performances will be used as references for character animation. To avoid the action getting too monotonous after reference, strive to intensify it. During this procedure, it is critical to pay attention to minor changes in action such as a head up, a hand up, and so on. When you are experiencing problems with animation creation, the easiest method to fix it is to do the movements in front of a mirror, evaluate them in detail, observe every movement, and try to exaggerate the action.

RETRACTED

During the animation of movement, the character's posture will change as a result of turning and shifting; the term “keyframe” refers to this changed posture. When creating keyframes, it is essential to accomplish the following goals: clear, contrast clear, and clear. The fluidity of the motion may be directly attributed to the quality of the keyframes, which are an integral part of any successful animation [15, 16]. First and foremost, in the process of production, a good keyframe action needs to be in sync with the performance of the character and the progression of the story. It should also be able to reflect the background, personality, and routines of the character, in addition to complying with the fundamental laws of motion and the equilibrium of forces. Then, a superb keyframe position must be appealing to the eye, in addition to being as exaggerated and engaging as is feasible. Finally, after drawing the keyframes, a trial run should be conducted to check whether the action conforms to the animation motion law. After confirming that the action is correct, the intermediate picture should be drawn, as shown in Figure 12. Lastly, after drawing the keyframes, a trial run should be conducted to check whether the action conforms to the animation motion law.

When it comes to animation, the law of motion is quite significant. This is due to the fact that simply having smooth movement is insufficient for animation creation. Exaggeration and comedy are two tools that may help us improve the eye-catching point in the animation process, which is what we need to do in order to accomplish what we need to accomplish, which is to get the audience's attention. Despite the fact that animation is derived from actual life, it is not the same as real life and must be exaggerated in order to accurately reflect reality. It will be less engaging if the characters in an animation walk and run in exactly the same way that people do in real life, because this will make the animation less realistic. In addition, while we are in the course of production, we need to record the action keyframes in order to give the characters a more tense appearance [17, 18].

RETRACTED

### 3.5. Postproduction Using the Intelligent Design Technology

To achieve the stunning visual performance that it is capable of, the animated short film must go through the postproduction process of cinema and television. Postproduction can save money that would otherwise be spent on filming and, in some cases, achieve results that filming cannot. As a result, postproduction synthesis may be regarded as a finishing touch. In postproduction, we first use After Effects (AE) to add special effects to the video, change the tone and light, and so on, in order to improve the overall texture of the short film. Then, we use surface light, parallel light, and other light sources to light the scene and give it color temperature. Then we export it and use PR to connect the dubbing and the images. Similarly, in order to ensure the good quality of the video, we will need to do numerous tests on the exported video to discover any errors and make the required modifications as soon as feasible. After completing all of the preceding processes, the created sequence is imported into After Effects and composited into a video, as shown in Figure 13.

To meet the film's postproduction standards, we had to render multiple scenes using layers, and we also incorporated a lot of special effects. The special effects portion of the animation was created using After Effects' effects plug-in, and a large number of the program's parameters were tweaked to achieve the desired animation effect. Following the completion of the visual effects work, the final color grading was done in accordance with the film's narrative, and the result was converted into an H.264 video file. The audio expression can help people believe that the shots are more seamlessly connected, which contributes to the overall impression that the short film is more harmonious and united. Animation combines audio and visual language. The next step is to do an overall color comparison in order to finish all of the elements that are visible and audible, as well as the output of the rendering.

## 4. Conclusion

The art of convergence media has entered people's lives and workplaces as cultural and creative industries continue to develop [19, 20]. In the age of convergence media, animation design is no longer limited to two-dimensional or three-dimensional creation, but has also given rise to a new form of animation expression known as MG animation. MG animation combines graphic design and a unique two-dimensional animation form, as well as formal movement style and design, to give the audience a unique experience. Despite the fact that MG animation has been around for decades, there are still some differences in academic circles regarding its definition. Some people believe that MG animation is the dynamic of static graphics and falls under the purview of graphic design. Another group believes that MG animation is a subset of animation because it possesses animation-like attributes and characteristics. To begin with, MG animation is a type of dynamic design derived from traditional static graphic design, with the characteristics, principles, and laws of traditional graphic design. Second, MG animation is used in dynamic media, such as animated advertisements and animated short films, where the time dimension expands and contracts. Finally, MG animation expands movement expression in time and space dimensions. MG animation is a graphic design product that uses an animation method and concept to create motion graphics, text, and symbols. Based on this context, it is of certain research value to examine the relevant elements of MG animation design and, in particular, the application of MG animation in the context of melting media. It is hoped that, by leveraging the benefits of convergence media, MG animation will exhibit greater permeability and interactivity, making message delivery more infectious. The animation created by the method described in this paper can also be used in the medical field for treatment management or lesion display.

RETRACTED

## Figures and Tables

**Figure 1:** Female owners.

**Figure 2:** Male leader.

**Figure 3:** Scene display 1.

**Figure 4:** Scene display 2.

**Figure 5:** Scene display 3.

**Figure 6:** Scene display 4.

**Figure 7:** Scene display 5.

**Figure 8:** Partial split script.

**Figure 9:** Main shot.

**Figure 10:** Animation process.

**Figure 11:** Character action binding.

**Figure 12:** Female running keyframe making interface.

**Figure 13:** After Effects' composite interface.

## Data Availability

The dataset used to support the findings of this study are available from the corresponding author upon request.
